The article "Nucleus Pulposus Cells Induce M2 Polarization of RAW264.7 via CX3CL1/CX3CR1 Pathway and M2 Macrophages Promote Proliferation and Anabolism of Nucleus Pulposus Cells" was retracted in 2024. Reasons: signs of a paper mill; suspected computer-generated content; unreliable results or conclusions; concerns about the data.

# Nucleus Pulposus Cells Induce M2 Polarization of RAW264.7 via CX3CL1/CX3CR1 Pathway and M2 Macrophages Promote Proliferation and Anabolism of Nucleus Pulposus Cells

**DOI:** 10.1155/2023/6400162

**Published:** 2023-02-20

**Authors:** Xiao-Tao Wu, Bo-Wen Wan, Xin-Min Feng, Yu-Ping Tao, Yong-Xiang Wang, Hui-Hui Sun

**Affiliations:** ^1^Spine Department, Northern Jiangsu People's Hospital, Yangzhou 225001, China; ^2^Spine Department, Zhongda Hospital, School of Medicine, Southeast University, Nanjing 210009, China

## Abstract

**Background:**

The mechanisms underlying M2 macrophage polarization induced by nucleus pulposus (NP) cells are unclear. The effects that M2-polarized macrophages have on NP cells are also controversial.

**Methods:**

Transcriptome sequencing was performed to detect the gene change profiles between NP cells from ruptured intervertebral disc (IVD) and normal IVD. The main difference on biological activities between the two cell groups were analyzed by GO analysis and KEGG analysis. Virus transduction, flow cytometry, immunofluorescence, RT-PCR, western blot, CCK-8, TUNEL staining, and AO/EB staining were performed to explore the interactions between NP cells and RAW264.7 macrophages. Statistics were performed using SPSS26.

**Results:**

801 upregulated and 276 downregulated genes were identified in NP cells from ruptured IVD in mouse models. According to GO and KEGG analysis, we found that the differentially expressed genes (DEG) were dominantly enriched in inflammatory response, extracellular matrix degradation, blood vessel morphogenesis, immune effector process, ossification, chemokine signaling pathway, macrophage activation, etc. CX3CL1 was one of the top 20% DEG, and we confirmed that both NP tissue and cells expressed remarkably higher level of CX3CL1 in mouse models (*p* < 0.001^∗^). Besides, we further revealed that both the recombinant CX3CL1 and NP cells remarkably induced M2 polarization of RAW264.7 (*p* < 0.001^∗^), respectively, while this effect was significantly reversed by si-CX3CL1 or JMS-17-2 (*p* < 0.001^∗^). Furthermore, we found that M2 macrophages significantly decreased the apoptosis rate (*p* < 0.001^∗^) and the catabolic gene levels (*p* < 0.001^∗^) of NP cells, while increased the viability, proliferation as well as the anabolic gene levels of NP cells (*p* < 0.01^∗^).

**Conclusions:**

Via regulating CX3CL1/CX3CR1 pathway, NP cells can induce the M2 macrophage polarization. M2 polarized macrophages can further promote NP cell viability, proliferation, and anabolism, while inhibit NP cell apoptosis and catabolism.

## 1. Introduction

Discogenic low back and leg pain contribute to severe movement disability globally [1] and is mainly caused by intervertebral disc (IVD) diseases [2]. The progression of IVD degeneration often begins with nucleus pulposus (NP) degeneration, which is the inner part of IVD and surrounded by annulus fibrosus and cartilage endplates. NP degeneration contains a complex of molecular and pathological changes and is generally characterized by the extracellular matrix degradation and resident cell apoptosis [3].

Healthy NP tissue is regarded as the immune privileged site [4]. Under degenerative condition, however, the immune cells are recruited into NP after the disruption of immunoinflammatory environment [4]. Previous studies have described that the presence of macrophages contributes to the deterioration of IVD degeneration, while these studies did not identify differentially polarized macrophages [5, 6]. As is well known, macrophages have good functional plasticity under certain pathological conditions. Recently, it has been revealed that M1 macrophages can promote IVD degeneration through aggravating extracellular matrix degradation and inducing apoptosis of NP cells [6]. Nevertheless, the interactions between M2 macrophages and NP cells have rarely been reported. Current findings on whether M2 macrophages promote the anabolism of NP cells or not are controversial [7, 8], indicating that more experiments are required to explore the crosstalk between M2 macrophages and NP cells. In addition, the mechanisms of M2 macrophage polarization in the NP tissue remain unknown.

Therefore, this research was performed to explore the mechanisms underlying M2 macrophage polarization induced by NP cells and to further reveal the effects that M2 macrophages have on NP cells.

## 2. Methods

### 2.1. Establishment of Mouse Models

Ethics approval was obtained for mice experiments from the Animal Care and Application Institute of the Research committee of Yangzhou University (yzu-lcyxt-n035), and all animal experiments were conducted based on the guidelines for the ethical treatment of animals of Yangzhou University.

C57BL/6 J mice (6 weeks; *n* = 6; male) were purchased from Comparative Medicine Centre of Yangzhou University. Mice were fixed in supine position on an operating table after anesthesia. A surgical incision was made along the abdomen midline after disinfection. Then, the viscera were gently pushed away until the L4-5 level of the spine was fully exposed. A 30G needle was inserted into the NP tissue at a depth of 2 mm for 2–3 times. Finally, the incision was sutured, and penicillin sodium was applied to prevent infection.

### 2.2. H&E Staining

On the 7th day after surgery, the lumbar spine was obtained and fixed with 4% paraformaldehyde for 24 h. After decalcification with EDTA for a month, the tissue was dehydrated, cleared, paraffinized, embedded, and finally sectioned (5 *μ*m thick). H&E Staining Kit (Hematoxylin and Eosin, ab245880) was utilized for staining to observe the histological features.

### 2.3. Immumohistochemical Staining

After deparaffinization and rehydration, Citrate Antigen Retrieval Solution (Beyotime, China) was used for antigen retrieval, followed by heating in a microwave for 5 min at 100°C. After the slides were cooled to room temperature, the slides were placed in 0.3% H_2_O_2_ for 10 min at room temperature. Incubate the slides with 5% goat serum for 10 min at room temperature. After that, add the primary antibody (RM80 for CD 80 and MR5D3 for CD206) at room temperature and incubate overnight. In the next day, secondary antibodies (anti-Rat IgG H&L, Alexa Fluor® 488 for RM80 and anti-mouse IgG–Peroxidase antibody, ThermoFisher for MR5D3) were added for 20 min at room temperature. 100 *μ*L DAB solution was dropped onto each slide under microscope. All slides were counterstained with hematoxylin and then washed in flowing tap water for 3 min. The samples were dehydrated, immersed in xylene, and finally were mounted.

### 2.4. Isolation of Nucleus Pulpous Cells

Mice were sacrificed by cervical dislocation. After disinfection with 75% alcohol, the mice were fixed on a supine position. The lumbar spine was separated under aseptic conditions, and then moved to the anatomical scope. The NP tissue was obtained and placed in DMEM/F12 culture medium containing 1% penicillin. Type 2 collagenase was added to digest the NP at 37°C for 1 h. Digestion was then terminated. Samples were centrifuged at 2000 r/min for 5 min. The complete medium was utilized to suspend the precipitate. Adjust the cell density to 1 × 10^5^ cells/mL. Then, the T25 square bottles were used to culture these cells. Put the bottles in an incubator (37°C, 5% CO_2_). Refresh the medium in half volume every 2 days. Cells were used for further experiment 5 days later. Only cells at logarithmic growth phase were selected for experiments in this study.

### 2.5. Preparation of RAW264.7 Macrophages

RAW264.7 (CX0022, BOSTER) was applied for this study. Cell density was adjusted to 1 × 10^5^ cells/mL. Aspirate 2 mL into the 6-well plates. Recombinant CX3CL1 (10 ng/ml) was added to treat the cells for 24 h to explore the efficiency of inducing M2 polarization, while JMS-17-2 (10 nmol/L, HY-123918, MCE) was used to detect that whether this effect can be reversed by inhibiting CX3CR1.

### 2.6. Establishment of Coculture System

RAW264.7 and NP cells adjusted the density of NP cells to 1.5 × 10^5^ cells/mL, and then 200 *μ*L was placed in the upper compartment of Transwell plate. Adjust Raw264.7 cell density to 8 × 10^5^ cells/mL, and then add 500 *μ*L in the lower chamber of Transwell plate (slide in advance).

M2 macrophages and NP cells was adjusted the NP cell density to 0.6 × 10^5^ cells/mL, and then 500 *μ*L was placed in the lower compartment of Transwell plate. Raw264.7 was treated by CX3CL1 for 24 h to obtain M2 macrophages. Adjust the cell density to 2 × 10^6^ cells/mL, and then put 200 *μ*L in the upper compartment of Transwell plate for 24 h.

### 2.7. Transcriptome Sequencing

NP cells of control group and model group were amplified and cultured in triplicate samples, and 5 × 10^6^ cells in each sample were collected. We discard the supernatant and add 1 ml Trizol to each sample. The samples were stored on dry ice and sent to Norhe source for transcriptome sequencing (supplementary material 1 for detailed information).

### 2.8. Immunofluorescent Staining

After the cells were treated for 24 h, the supernatant on the slides was aspirated, and 100 *μ*L of 4% paraformaldehyde was used for fixation for 30 min. Remove the fixation solution and wash the cells. Add 100 *μ*L 0.1% Triton x-100 to each slide at room temperature for 3 min. Add 300 *μ*L 5% BSA blocking solution to each slide and put the slides in an incubator (5% CO_2_, 37°C) for 1 h. Wash with PBS and aspirate the liquid. Add 100 *μ*L to each slide, and use 1% BSA diluted CX3CL1 (1 : 500) or F4/80 (1 : 500) or CD206 (1 : 1000). Incubate the slides at 4°C overnight. Add 100 *μ*L PBS to each slide for 5 min and aspirate the liquid, repeat 3 times. Add 100 *μ*L 1% BSA blocking solution to each slide for 15 min at room temperature. Add 100 *μ*L to each slide with 1% BSA diluted CY3-labeled Donkey anti-rabbit IgG (1 : 100), and incubate at 37°C for 1 h. Add 100 *μ*L PBS to each slide for 5 min and aspirate the liquid, repeat 3 times. Add 100 *μ*L Hoechst33258 dye solution to each slide, and incubate for 10 min at room temperature away from light. The slides were then sealed with anti-fluorescence quenching sealing solution. Finally, the slides were photographed under fluorescence microscope.

### 2.9. Reverse Transcription-Polymerase Chain Reaction (RT-PCR)

Total RNA was extracted using TRIzol reagent method (Takara, Japan) following the manufacturer's protocols. RNA (2 *μ*g) was converted into cDNA using RevertAid First Strand cDNA Synthesis Kit (Thermo, Shanghai). Primer Premier 5.0 (Sangon Biotech, Shanghai) was used to design gene primers (Table 1). The PCR reaction was performed as the following procedures: 95°C for 5 min, then followed by 40 cycles of 10s at 95°C and 30s at 60°C. *β*-Actin was chosen as the internal reference gene. The relative gene expression levels were calculated using 2^−*ΔΔ*Ct^ method.

### 2.10. Western Blot

Collect the cells after treatment for 7 days. 200 *μ*l of RIPA lysis buffer and an appropriate amount of PMSF was added. The cells were lysed on ice for 2 h. Centrifuge cells at 12,000 r/min for 10 min at 4°C. After that, transfer the supernatant to a new EP tube. Bicinchoninic Acid (BCA) Kit (Thermo, Shanghai) was used for protein quantification. Prepare 12% separation gel and 5% concentrated gel in advance. Proteins were added into 200 *μ*l EP tubes. Add 3 *μ*l dye solution to each tube. Protein denaturation was conducted at 95°C for 5 min. 30 *μ*g protein was added to each well. SDS-PAGE electrophoresis was performed (80 V, 20 min for concentrated gel; 120 V, 1 h for separation gel). Transfer the membrane. Place the membrane into 5% BSA solution at room temperature for 1 h. Separately add the primary antibody of Rabbit monoclonal anti-CX3CL1 (DF12376, Affinity, 1 : 500) and Mouse monoclonal anti-actin (GB11001, Servicebio, diluted at 1 : 2000). Keep the membranes in a refrigerator at 4°C overnight. In the next day, wash the membranes with TBST for 5 times. The second antibody was added for 1 h at 37°C. Wash the membranes again with TBST for 5 times. Visualization was conducted using enhanced chemiluminescence (ECL) luminescent liquid.

### 2.11. Flow Cytometry

To detect the proportion of M2 macrophages, centrifuge tubes at 1500 r/min for 5 min to collect macrophages. Resuspend the cells with precooling PBS (4°C). Centrifuge cells at 1500 r/min for 5 min. Add 300 *μ*L of 1^∗^Binding Buffer to suspend the cells. 5 *μ*L F4/80 and 0.25 *μ*L CD206 were added to stain the cells. Mix the tubes well and incubate for 15 min at room temperature away from light. After washing, add 300 *μ*L Binding Buffer before delivering to flow cytometry.

To explore the NP cell apoptosis rate, digest and collect NP cells using trypsin digestion without EDTA. Centrifuge the samples at 1500 r/min for 5 min. Resuspend NP cells with precooling PBS (4°C). Centrifuge at 1500 r/min for 5 min, and then wash cells. Add 300 *μ*L of 1^∗^Binding Buffer to suspend cells. Add 10 *μ*L Annexin V-FITC and 5 *μ*L PI for staining. Mix well. Put the mixture at room temperature away from light for 15 min. Wash cells. Add 400 *μ*L Binding Buffer before delivering to flow cytometry.

### 2.12. siRNA Transfection

Negative control (NC) and Si-CX3CL1 (75 pmol, sense: GCUGUGGCAGUAACUCAUATT; antisense: UAUGAGUUACUGCCACAGCTT) was diluted with 100 *μ*L serum-free medium. Mix Lipofectamine2000 gently before use. Then, dilute 12 *μ*L Lipofectamine2000 with 100 *μ*L serum-free DMEM. Incubate cells for 5 min at room temperature. Add liquid A and B and gently mix well. Incubate cells at room temperature for 15 min to form the transfection complex. The supernatant was aspirated from the 6-well plates. 1800 *μ*L serum-free medium was added to each well. Add 200 *μ*L of the mixture to each well, and put the plate in an incubator (5% CO_2,_ 37°C) for 6 h. Then, aspirate the supernatant and add 2 mL of complete medium. Collect the cells for further experiments after 48 h.

### 2.13. Cell Viability Assay

After 48 h of culture, add 200 *μ*L of CCK8 solution (Dojindo, Japan) to each well in lower chamber. Incubate cells in an incubator (5% CO_2_, 37°C) for 2 h away from light. The OD value was measured using a microplate reader (CliniBio 128, Austria) at a wavelength of 450 nm and was used to further calculate the cell viability.

### 2.14. TUNEL Staining

TUNEL staining kit (Beyotime Biotech) was used the following protocols. Wash NP cells with PBS and fix them for 30 min with fixation solution (P0098, Beyotime Biotech). Wash again with PBS. Put cells in strong permeable solution (P0097, Beyotime Biotech) and incubate for 5 min at room temperature. Prepare TUNEL detection solution: 25 *μ*L TdT enzyme +225 *μ*L fluorescent labeling solution +250 *μ*L TUNEL detection solution. Add 50 *μ*L TUNEL detection solutions to the samples. Put the samples away from light for incubation at 37°C for 60 min. Wash with PBS for 3 times, then add Hoechst (C1017, Beyotime Biotech) for staining for 10 min. Wash with PBS for 3 times. Anti-fluorescence quenching solution was used to seal the slides before observation.

### 2.15. AO/EB Staining

AO/EB staining kit (BestBio, China) was applied to explore the survival status of NP cells. Staining and incubation was performed following the protocols. 10 *μ*l of cell suspension was placed on a microslide and then observed under a fluorescence microscope.

### 2.16. Statistics

SPSS version 26 (IBM Corp., USA) was applied for statistics. The continuous variables were shown as the mean values ± standard deviation. Statistically significant difference was evaluated using a *t*-test between two groups. A p < 0.05 at 2 sides was used to represent a significant difference. In addition, *p* − adjust (p.adj) < 0.05 was used to represent a significant difference for bioinformatics analysis.

## 3. Results

### 3.1. Quality Control of Transcriptome Sequencing

To clarify the overall gene changes between NP cells from ruptured IVD models (M group) and normal NP cells (N group), transcriptome sequencing was performed which involved 3 samples in each group. The raw data were uploaded in the NCBI database (PRJNA852654). An average of 44866651 and 45476432 raw reads were generated for each sample in M group and N group, respectively. Only 43072377 and 43553840 clean data with high quality, which represented 96.0% and 95.8% of total reads for each group, were obtained for analysis. The Q20 values were 97.6% and 97.7% for M group and N group (supplementary material 2). The error rates ranged from 0.02% to 0.04% for each sample in both groups (supplementary material 3). The level of bases (A/T and G/C contents) was stable for each sample (supplementary material 4). Besides, the FPKM values were comparable across different samples in each group (supplementary material 5). The Pearson correlation coefficient between samples was extremely high, with *R*^2^ > 0.86 in M group and *R*^2^ > 0.97 in N group (supplementary material 6). Moreover, we found that exons accounted for more than 80% of genome regions in each sample of both groups (supplementary material 7). The above results indicated that the quality of our sequencing is extremely high.

### 3.2. Differentially Expressed Genes and Differential Molecular Profiling

Overall, 11815 overlapped genes were identified for the two groups (Figure 1(a)), with 801 upregulated and 276 downregulated genes in M group (Figure 1(b)). Clustering of differentially expressed gene data as well as the similarities and differences among samples were presented in the heatmap (Figure 1(c)).

Further, according to GO and KEGG analysis, we revealed the differentially biological activities between the two groups. A total of 42 pathways were downregulated and 1090 pathways were upregulated in M group according to GO analysis (supplementary material 8), while only 4 pathways were downregulated and 42 pathways were upregulated in N group according to KEGG analysis (supplementary material 8). Significantly enriched biological processes in GO analysis included inflammatory response, extracellular matrix, blood vessel morphogenesis, immune effector process, ossification, and so on (Figure 2). Significantly enriched pathways in KEGG analysis mainly contained chemokine signaling pathway, PI3K-Akt signaling pathway, etc. (Figure 3).

CX3CL1 was in the top 20% differentially expressed genes in this study (Figure 1(c)) and was significantly involved in a few biological activities, such as cytokine receptor binding, inflammatory response (Figure 2), and chemokine signaling pathway (Figure 3). Since CX3CL1 and its exclusive receptor CX3CR1 can induce M2 macrophage polarization in cancer settings [9], CX3CL1 was selected as the target gene to further explore whether NP cells can induce M2 macrophage polarization in degenerated IVD in this study.

### 3.3. Presence of M2 Macrophages and CX3CL1/CX3CR1 in the Intervertebral Disc

The herniated IVDs were entirely obtained from mouse models at 2 weeks after surgery, while controlled specimens were obtained from healthy mice (*n* = 3, Figure 4(a)). Herniated IVD contained much more M1 (*n* = 3, Figure 4(b)) and M2 (*n* = 3, Figure 4(c)) macrophages than normal IVD. These infiltrated macrophages distributed both in the outer layer of annulus fibrosus and the inner NP tissue (Figures 4(b) and 4(c)). Only interactions between NP cells and M2-polarized macrophages were explored in this study.

Besides, we revealed that CX3CR1 was positively stained in almost all M2 macrophages in degenerated NP tissue (Figure 5(a)). Moreover, NP tissue from herniated IVD expressed significantly higher level of CX3CL1 (*p* < 0.001, Figures 5(b)–5(d)).

### 3.4. Nucleus Pulposus Cells Induce M2 Polarization of Macrophages through CX3CL1/CX3CR1 Axis

To explore the interactions between CX3CL1 and macrophages, recombinant CX3CL1 was applied to treat RAW264.7. CX3CL1 remarkably induced M2 polarization of RAW264.7 (*p* < 0.001, Figure 6), while this effect was measurably reversed by JMS-17-2 (*p* < 0.001, Figure 6), which is an inhibitor of CX3CR1.

Further, the coculture chamber of RAW264.7 and NP cells was established (Figure 7(a)). After coculture for 24 h, NP cells dramatically produced higher CX3CL1 level than those NP cells cultured alone (*p* < 0.001, Figures 7(b)–7(d)). Meanwhile, the proportion of M2 macrophages significantly rose up in the coculture system (*p* < 0.001, Figures 7(e)–7(h)), indicating that NP cells can induce M2 polarization of RAW264.7.

Moreover, we designed three siRNAs to detect their efficiency in silencing CX3CL1 and found that siRNA-3 was most efficient (Figure 8(b)), which was named si-CX3CL1 and was used for further experiments. Four groups were set to explore the effects of CX3CL1 in the process of NP cell induced M2 macrophage polarization: RAW264.7 alone, RAW264.7 + NP cells+si-NC, RAW264.7 + NP cells+si-CX3CL1, and RAW264.7 + NP cells+JMS-17-2. We revealed that NP cells significantly induced M2 polarization of RAW264.7 (*p* < 0.001, Figure 8), while both si-CX3CL1 and JMS-17-2 significantly decreased the efficiency in M2 polarization of RAW264.7, respectively (*p* < 0.001, Figure 8). The results indicated that silencing CX3CL1 or CX3CR1 can prevent the M2 polarization of RAW264.7 induced by NP cells.

### 3.5. Effect of M2 Macrophages on Nucleus Pulposus Cells

Recombinant CX3CL1 was used to treat RAW264.7 to obtain M2 macrophages, which were further cocultured with NP cells. We found that M2 macrophages significantly reduced the apoptosis rate of NP cells (*p* < 0.001, Figures 9(a), 9(b), and 9(d)) and promoted the viability of NP cells (*p* < 0.001, Figure 9(c)). Besides, we revealed that M2 macrophages significantly promoted the PCNA level in NP cells, while the ratio of BAX/Bcl-2 genes reduced dramatically (*p* < 0.001, Figure 9(e)), which indicated that M2 polarized macrophages promoted the NP cell proliferation. Furthermore, we found that M2 macrophages significantly promoted COL-2 and ACAN levels (*p* < 0.001, Figure 9(f)), while reduced TNF-*α*, IL-6 and MMP-3 levels (*p* < 0.001, Figure 9(f)) in NP cells, indicating that M2 macrophages inhibited the degradation of extracellular matrix.

## 4. Discussion

IVD has long been recognized as the immune privileged tissue, and it can attract the macrophages upon the breakdown of immune microenvironment during degeneration process [4]. Nevertheless, the interactions between NP cells and macrophages are rarely studied. Transcriptome analysis in earlier studies did not focus on the changes related to immune response. Biological changes in ruptured IVD are different from that in contained IVD due to more severe immune response [4]. However, the differentially expressed gene profiles between NP cells in ruptured IVD and normal IVD have seldom been reported. Therefore, in this study, we revealed that apart from inflammation response and extracellular matrix degradation, genes related to chemokine signaling pathways, immune response, and macrophages activation were also significantly enriched through GO and KEGG analysis.

Previous studies have demonstrated that M1 macrophages can accelerate the IVD degeneration [5], while the effects that M2 macrophages have on NP cells are still not well understood, and available outcomes are inconsistent [7, 8]. Here we described the differentially expressed gene profiles and main biological processes in NP cells from ruptured IVD. Besides, we further reported that NP cells induced M2 polarization of macrophages via CX3CL1/CX3CR1 axis, and M2 macrophages promoted the NP cell proliferation and viability and inhibited the cell apoptosis and degradation of extracellular matrix.

The only one member of the CX3C chemokine family is CX3CL1, which specifically binds to the receptor CX3CR1 [10]. High CX3CL1 level is strongly related to IVD degeneration and radicular pain, with degenerated NP produced more CX3CL1 [11]. Besides, another study revealed that herniated NP tissue expressed significantly higher level of CX3CL1 and CX3CR1 [12]. This is consistent with our findings. CX3CR1 is mainly expressed on immune cells, such as monocytes and macrophages, and CX3CL1 is chemotactic for these cells [13]. In addition, T cells and NK cells also contribute to IVD degeneration through expressing CX3CR1 [12]. Early researches have showed that CX3CL1-CX3CR1 axis tends to induce M2 macrophage polarization in many other diseases [9, 14], and deficiency of CX3CR1 resulted in a decrease of M2 macrophage infiltration and a reduction of collagen level [15]. However, the role of CX3CL1/CX3CR1 axis in the M2 macrophage polarization during IVD degeneration is still unknown. In this study, we revealed that degenerated NP tissue expressed significantly higher CX3CL1 than normal NP, and this is consistent with the outcomes of other studies [11, 16]. Besides, we further revealed that majority of infiltrated M2 macrophages strongly expressed CX3CR1, and both recombinant CX3CL1 and NP cells significantly induced M2 polarization of RAW264.7. While this effect was totally reversed by si-CX3CL1 or JMS-17-2, which has been frequently used as an inhibitor of CX3CR1 [17], indicating that CX3CL1/CX3CR1 axis was involved in the recruitment of M2 macrophages in the degenerated NP tissue.

On the other hand, Fas ligand (FasL), which acts as maintaining the immune privilege [18], is also highly expressed on NP cells [19]. It has been reported that NP cells can prevent angiogenesis [20] and infiltration of macrophages and T cells [21] via regulating FasL-mediated cell apoptosis. Yet the expression of FasL significantly decreased in degenerated IVD [19]. Besides, a previous study has reported that CX3CL1-CX3CR1 axis serves as maintaining cell survival and inhibiting FasL-induced cell death [22]. This may at least partly explain the persistence of macrophages in the ruptured IVD, especially in NP tissue.

Some studies declared that the infiltrating macrophages may enhance the inflammatory conditions in degenerated IVD [5] and reduced the expression of ACAN and COL-2 to aggravate the loss of extracellular matrix [6]. Indeed, M1 macrophages promote the extracellular matrix degradation and reduce NP cell viability, and finally lead to the progression of IVD degeneration [5, 23]. However, the effects that M2 macrophages have on NP cells are controversial.

The presence of M2 macrophages in the ruptured IVD has been occasionally reported recent years [7, 8, 24]. It has been declared that the M2 macrophages were differentiated from resident macrophages in IVD and were regulated by TGF-*β* [24], while another study reported that M2a macrophages were absent in normal IVD but recruited in degenerated IVD in mice [7]. The above contrary findings indicate that the origin of M2 macrophages in IVD is still unclear. Besides, the study also revealed that M2a macrophages decreased the expression of ACAN and COL-2 and improved the MMP-3 and MMP-9 levels in NP cells via regulating CHI3L1/IL-13Ra2 pathway [7]. In addition, another study reported that M2 macrophage-conditioned medium can prevent IVD degeneration through promoting the proliferation of NP cells, inhibiting inflammation, cell apoptosis, and senescence as well as enhancing the expression of COL-2 and ACAN [8]. These inconsistent findings further indicate that the effects that M2 macrophages have on NP cells are still debatable. In the present study, we found that M2 macrophages reduced NP cell apoptosis and increased their viability and proliferation. In addition, we further confirmed that M2 macrophages improved the expression level of COL-2 and ACAN, while inhibited the level of TNF-*α*, IL-6, and MMP-3 in NP cells, indicating that M2 macrophages act as contributing to the repair of the extracellular matrix.

## 5. Conclusions

The presence of M2 macrophages in degenerated IVD has long been noticed. In this study, we revealed the biological processes related to IVD degeneration, including inflammation response, extracellular matrix degradation, immune effector process, chemokine signaling pathway, and macrophage activation. Besides, we also found that NP cells induced M2 polarization of macrophages via CX3CL1/CX3CR1 axis, while M2 macrophages further promoted the NP cell proliferation and viability and inhibit the NP cell apoptosis and extracellular matrix degradation. Our findings support the strategy that promoting the polarization of macrophages to an anti-inflammatory M2 phenotype can improve the poor healing capacity of degenerated IVD [25].

## Figures and Tables

**Figure 1:** M group and N group represent nucleus pulposus cells isolated from ruptured IVD and normal IVD, respectively. (a) Totally 11815 genes were coexpressed in both groups, (b) among which 801 were upregulated and 276 were downregulated. (c) Heatmap of differentially expressed genes between the two cell groups with 3 samples in each group.

**Figure 2:** GO analysis found that differentially expressed genes were significantly enriched in many biological activities, such as inflammatory response, blood vessel morphogenesis, and immune effector process. CX3CL1 was involved in inflammatory response, receptor regulator activity, etc. Only top 10 terms in BP, CC and MF were presented. “^∗^” indicates a *p*.adj < 0.05. “#” indicates that CX3CL1 was involved in the process. BP: biological process; CC: cell component; MF: molecular function.

**Figure 3:** KEGG analysis found that differentially expressed genes were significantly enriched in many pathways, including PI3K-Akt pathway, Rapl signaling pathway, and chemokine signaling pathway. CX3CL1 was involved in chemokine signaling pathway. Only top 20 enriched pathways were presented for upregulated genes and down regulated genes, respectively. “^∗^” indicates a p.adj < 0.05. “#” indicates that CX3CL1 was involved in the process.

**Figure 4:** H&E staining showed that the IVD in mouse models herniated into the spinal canal. In comparison with the normal IVD, it was clear that the height of IVD space became narrow, the shape of NP tissue became sharp, the annulus fibrosus became thinned and damaged, and the extracellular matrix was also degenerate in the mouse models. These changes altogether indicated that the IVD was severely degenerated in mouse models (a). IHC staining showed that measurable amounts of CD80+M1 and CD206+M2 macrophages (brown color) infiltrated in herniated IVDs, while no macrophages presented in normal IVD (b, c). Further we found that these infiltrated macrophages (brown color) mainly distributed in the outer layer of annulus fibrosus, and the inner degenerated NP tissue (b, c).

**Figure 5:** Almost all CD206+M2 macrophages expressed high level of CX3CR1 (a). RT-PCR (b) and immunofluorescent staining (c, d) confirmed that degenerated NP tissue expressed significantly higher level of CX3CL1. “^∗∗∗^” indicates *p* < 0.001. IVD: intervertebral disc. NP; nucleus pulposus.

**Figure 6:** Recombinant CX3CL1 significantly increased the proportion of M2 macrophages, while this effect was reversed by adding JMS-17-2 as measured by immunofluorescent staining (a) and flow cytometry (b). “^∗∗∗^” indicates *p* < 0.001. RAW: RAW264.7 macrophages.

**Figure 7:** NPC were spindle in shape and were able to adhering to the wall, while the RAW264.7 macrophages were round in shape, well clustered, and also able to adhering to the wall (a). In the coculture system, RAW264.7 significantly increased the expression of CX3CL1 in NPC (b–d). Besides, NPC significantly induced M2 polarization of RAW264.7 as measured by flow cytometry (e, f) and immunofluorescent staining (g, h). “^∗∗∗^” indicates *p* < 0.001. RAW: RAW264.7 macrophages. NPC: nucleus pulposus cells.

**Figure 8:** Three siRNAs were designed. It turned out that the siRNA-3 (named si-CX3CL1) showed the highest efficiency and was selected for the further experiment (b). si-CX3CL1 and JMS-17-2 significantly suppressed the M2 polarization of RAW264.7 induced by NPC as measured by immunofluorescent staining (a, c) and flow cytometry (f, e). “^∗∗∗^” indicates *p* < 0.001, “^∗∗^” indicates *p* < 0.01. RAW: RAW264.7 macrophages. NPC: nucleus pulposus cells.

**Figure 9:** Coculture system of M2 macrophages and NPC was established. M2 macrophages reduced the apoptosis rate of NPC although did not reach a significant level as measured by TUNEL staining (a). However, the reduction of apoptosis rate reached the significant level in AO/EB staining assay (b) and flow cytometry (d). CCK-8 assay revealed that M2 macrophages significantly increased the NPC viability (c). Meanwhile, the expression level of PCNA gene increased, and the ratio of Bac/Bcl-2 genes decreased in NPC (e). Moreover, the expression level of COL-2 and ACAN significantly increased in NPC, while the expression level of TNF-*α*, IL-6, and MMP-3 significantly decreased in NPC (G). “^∗∗∗^” indicates *p* < 0.001, “^∗∗^” indicates *p* < 0.01. “^∗^” indicates *p* < 0.05. RAW: RAW264.7 macrophages. NPC: nucleus pulposus cells.

**Table 1:** Primers of the genes in this study.

Genes	Primers	Sequences
PCNA	Forward primer	5′-CTTCTTCACGGTTGCAGGGA-3′
	Reverse primer	5′-ATTCACCCGACGGCATCTTT-3′
BAX	Forward primer	5′-CTGGATCCAAGACCAGGGTG-3′
	Reverse primer	5′-CCTTTCCCCTTCCCCCATTC-3′
Bcl-2	Forward primer	5′-AGCATGCGACCTCTGTTTGA-3′
	Reverse primer	5′-GCCACACGTTTCTTGGCAAT-3′
COL-2	Forward primer	5′-GCGACCGGGAGCATATAACT-3′
	Reverse primer	5′-GCCCTAATTTTCGGGCATCC-3′
ACAN	Forward primer	5′-CATGCTTATGCCTTCCGAGC-3′
	Reverse primer	5′-CTTTCTTCTGCCCGAGGGTT-3′
TNF-*α*	Forward primer	5′-ACCCTCACACTCACAAACCA-3′
	Reverse primer	5′-ACCCTGAGCCATAATCCCCT-3′
IL-6	Forward primer	5′-CACAAGTCCGGAGAGGAGAC-3′
	Reverse primer	5′-TTGCCATTGCACAACTCTTT-3′
MMP-3	Forward primer	5′-CATCCCCTGATGTCCTCGTG-3′
	Reverse primer	5′-CTTCTTCACGGTTGCAGGGA-3′
*β*-Actin	Forward primer	5′-TATTGGCAACGAGCGGTTCC-3′
	Reverse primer	5′-GCACTGTGTTGGCATAGAGG-3′

## Data Availability

All the data in this study are available from the corresponding author on reasonable request.

## Abbreviations

IVD: Intervertebral disc
NP: Nucleus pulposus.

## Supplementary Materials

Supplementary 1 Supplementary Material 1. Methods of transcriptome sequencing and data analysis.

Supplementary 2 Supplementary Material 2. Original table and figures presenting clean reads and Q20 values.

Supplementary 3 Supplementary Material 3. Original figures presenting error rates for the samples.

Supplementary 4 Supplementary Material 4. Original figures presenting A/T and G/C contents for the samples.

Supplementary 5 Supplementary Material 5. Original table presenting FPKM values for the samples.

Supplementary 6 Supplementary Material 6. Original table and figures presenting the Pearson correlation coefficient between samples.

Supplementary 7 Supplementary Material 7. Original figures presenting the percentages of exons for the samples.

Supplementary 8 Supplementary Material 8. All significantly enriched biological activities and pathways obtained via GO and KEGG analysis.
